# Analysis of 78 Cases of Primary Gastrointestinal Lymphoma

This article has been retracted.

**DOI:** 10.1155/2022/3414302

**Published:** 2022-03-19

**Authors:** Yu Xiang, Lidi Yao

**Affiliations:** ^1^Department of Gastroenterology, Huzhou Central Hospital, Huzhou, China; ^2^Department of Radiology, Huzhou Central Hospital, Huzhou, China

## Abstract

This paper studied the pathological features of 78 cases of primary gastrointestinal lymphoma. All patients with primary gastrointestinal lymphoma diagnosed in PET Center of Zhebei Mingzhou Hospital in Huzhou from August 2013 to April 2021 were analyzed retrospectively. In addition, the pathology and immunohistochemistry of these patients were retrieved from the inpatient system of Huzhou Central Hospital. The results showed that the male-female ratio of these 78 patients was about 1.29/1 (including 44 males and 34 females), with a median age of 63 years old (20–90 years old). The most frequent sites in order of its occurrence were the stomach (51.3%), small intestine (34.6%), ileocecal region (9%) and colon (5.1%). T-cell lymphoma accounted for 10.7% of primary gastrointestinal lymphoma, and all of them were found in small intestines, while B-cell lymphoma accounted for 89.3%.

## 1. Introduction

Primary gastrointestinal lymphoma (PGIL) is a malignant tumor originating from the submucosal lymphoid tissue of the gastrointestinal tract and is the most common extranodal lymphoma, accounting for about 30%–40% of all extranodal lymphomas and 4% of gastrointestinal tumors. PGIL may occur in the whole digestive tract, and the stomach is the most commonly involved site (60%–75%) in the gastrointestinal tract followed by small intestine (20%–30%), large intestine (5%–10%) and esophagus (<1%) [1–3]. In general, the majority of all gastrointestinal lymphomas are B-cell lymphomas, whereas T-cell lymphoma is less common, accounting for only 6% [3]. The affected patients are usually at the age between 50 and 70 years old [4, 5]. Most patients have overlapping symptoms of other gastrointestinal diseases, without specific manifestations under endoscopy. Therefore, histopathological examination is prerequisite for determining diagnosis [6]. However, the best way to obtain pathology is through endoscopic biopsy. Endoscopic biopsy is extremely important for the diagnosis of this disease, but in clinic, biopsy lymphoma is often negative. Possible reasons are as follows: (1) Tumor tissue in lamina propria of mucosa is softer than cancer tissue, which is easy to be damaged during biopsy, the location of autolysis sample is inaccurate and the depth is not enough; (2) The collected tissue cannot clearly show the glandular duct tissue, which is not easy to distinguish from poorly differentiated adenocarcinoma; (3) Early lesions were located in submucosa and infiltrated downward, the mucosa was intact, the lesion could not be located under endoscope, and the biopsy depth was not enough, so it was difficult to get the lesion tissue.

Pathogenesis of primary gastrointestinal lymphoma: (1) immune causes: like most malignant tumors, the immune surveillance system is too low, which easily leads to the occurrence of tumors. (2) Microbial infection: at present, it is generally accepted that the occurrence of MALT lymphoma in the stomach is closely related to *Helicobacter pylori* infection.

Clinical staging is very important for the treatment of primary gastrointestinal lymphoma and the prognosis evaluation of patients. Most malignant tumors have corresponding clinical staging to guide the diagnosis and treatment of patients. However, there is no recognized staging method for primary gastrointestinal lymphoma. At present, the common clinical staging methods are Musshoff, Ann Arbor and Lugano. Lugano staging standard, which was introduced in 2014, is widely used in clinical trials and clinical practice, and is used for response evaluation of lymphoma.

In this paper, 78 patients with lymphoma were analyzed by age, sex, sites, pathological features and immunohistochemical analysis, with the purpose of gaining a deeper understanding of this disease.

## 2. Materials and Methods

### 2.1. Case Data

The paper studied patients diagnosed with primary gastrointestinal lymphoma in Huzhou Central Hospital from August 2013 to April 2021. Among the 78 patients, there were 45 males and 34 females, with a male-female ratio of about 1.29/1. The age ranged from 20 to 90 years old, with a median age of 63 years old. All cases were diagnosed by imaging. In addition, the pathology and immunohistochemistry of these patients were retrieved from the inpatient system of Huzhou Central Hospital. Among them, 56 cases were confirmed by pathological biopsy, including histopathological and immunohistochemical diagnosis. The information of sex, age and pathological types of 78 patients were collected, and the corresponding characteristics were analyzed.

### 2.2. Pathological Classification and Diagnostic Criteria

Pathological classification of 79 patients was referred to WHO Classification of Tumors of Haematopoietic and Lymphoid Tissue issued in 2016. The diagnostic criteria follow that proposed by Dawson [7]: (1) no pathological enlarged superficial lymph nodes; (2) no enlarged mediastinal lymph nodes; (3) normal count and classification of WBC; (4) surgery confirms that the lesion originates in the gastrointestinal tract, and no other masses are found except lymph nodes involved in drainage area and surrounding organs directly invaded; (5) normal liver and spleen.

In addition, other examinations can be performed to exclude the existence of extraintestinal lymphomas.

## 3. Results

### 3.1. General Information

#### 3.1.1. Gender Distribution

The gender analysis of 78 patients showed that the PGIL incidence of males was higher than that of females, where males account for about 56% and females account for 44%. Gender distribution is shown in Figure 1.

#### 3.1.2. Age Distribution

The age range of these 78 patients is 20–90 years old, with an average age of about 61.16 years old and a median of 63 years old, suggesting that the incidence of PGIL reaches its peak among middle-aged and elderly people.See Figure 2 for age distribution.

### 3.2. Clinical Manifestations

#### 3.2.1. Sites of Incidence of Primary Gastrointestinal Lymphoma

The most frequent sites in order of occurrence of PGIL are the stomach (51.3%), small intestine (34.6%), ileocecal region (9%) and rectum and colon (5.1%). See Figure 3 for the sites of incidence.

There were 40 cases (51.3%) of Primary Gastrointestinal Lymphoma in the stomach, 27 cases (34.6%) in the small intestine, 7 cases (9%) in the ileocecal region, and 4 cases (5.1%) in rectum and colon. There was no data for primary esophageal lymphoma due to the small sample and the extremely low incidence of primary esophageal lymphoma.

### 3.3. Histopathological Features of Primary Gastrointestinal Lymphoma

#### 3.3.1. Pathological Features

Histopathological specimens were obtained from 56 cases of primary gastrointestinal lymphoma by operation, endoscopy, B-ultrasound or CT guided puncture, including 56 cases of non-Hodgkin's lymphoma and 0 cases of Hodgkin's lymphoma. Among non-Hodgkin's lymphomas, 49 cases were B-cell lymphoma, accounting for 87.5%, and 7 cases were T-cell-derived lymphoma, accounting for 12.5%.

Among 49 cases of B-cell lymphoma, there were 42 cases of diffuse large B-cell lymphoma (about 85.8%), 4 cases of MALT lymphoma (about 8.2%), 1 case of mantle cell lymphoma (about 2%), 1 case of follicular lymphoma (about 2%), and 1 case of B-lymphoblastic lymphoma (about 2%). See Figure 4 for case distribution.

### 3.4. Pathological Features of Lymphoma at Different Sites

#### 3.4.1. Pathological Analysis of Gastric Lymphoma

Diffuse large B lymphoma is the most common type of gastric lymphoma, with the incidence rate accounting for nearly 80% (24 cases), followed by MALT lymphoma (4 cases, about 13.3%), mantle cell lymphoma (1 case, about 3.3%). Due to the small sample, there are only three types of lymphoma in the stomach. See Figure 5 for the distribution of gastric lymphoma.

#### 3.4.2. Pathological Analysis of Small Intestinal Lymphoma

The pathological cases of lymphoma in small intestine (including terminal ileum) in order were diffuse large B-cell lymphoma (9 cases, about 50%), NK/T-cell lymphoma (7 cases, about 38.8%), follicular lymphoma (1 case, about 5.6%) and B-lymphoblastic lymphoma (1 case, about 5.6%). Among lymphomas occurring in the small intestine, the incidence of T-cell-derived lymphoma was higher than that of other sites. In this sample, almost all cases of NK/T-cell-derived lymphoma were found in the small intestine. In addition, there was a case of B-lymphoblastic lymphoma, a 29-year-old male with high-grade malignancy. See Figure 6 for the distribution of small intestinal lymphoma.

#### 3.4.3. Pathological Analysis of Ileocecal Lymphoma

The pathology of ileocecal lymphoma was diffuse large B-cell lymphoma.

#### 3.4.4. Pathological Analysis of Colorectal Lymphoma

The pathology of colorectal lymphoma was diffuse large B-cell lymphoma.

### 3.5. Specific Analysis

#### 3.5.1. Epidemiological Characteristics of Primary Gastrointestinal Lymphoma

Primary gastrointestinal lymphoma accounted for about 30%–40% of all extranodal lymphomas and 4% of gastrointestinal tumors. PGIL may occur in the whole digestive tract, and the stomach is the most commonly involved site (60%–75%) in the gastrointestinal tract followed by small intestine(20%–30%), large intestine (5%–10%) and esophagus (<1%) [1–3]. In general, the majority of all gastrointestinal lymphomas are B-cell lymphomas, whereas T-cell lymphoma is less common, accounting for only 6% [3]. In this study, gastric lymphoma accounted for about 50.1%, which was lower than the reported proportion. The possible reason, the author speculates, lies in the fact that some patients are not admitted to the ward. The sample objects of this study are mainly inpatients, and some patients with gastric lymphoma suffer from indolent gastric MALT lymphoma, which may be routinely treated with anti-Helicobacter pylori medicine in the outpatient department. Therefore, they are not admitted to the ward for hospitalization. It is widely recognized that diffuse large B-cell lymphoma is the most common pathological type of lymphoma, followed by MALT lymphoma. In this study, all NK/T cell-derived lymphomas were found in the small intestine.

#### 3.5.2. Primary Gastric Lymphoma

Gastric diffuse large B-cell lymphoma is the most common pathological type of gastric lymphoma. About 40% of primary gastric lymphoma is indolent lymphoma, among which gastric mucosa-associated lymphoid tissue (MALT) lymphoma is the most common one, followed by follicular lymphoma, Burkitt lymphoma and mantle cell lymphoma.

#### 3.5.3. Primary Gastric MALT Lymphoma

In this study, there were not many cases of gastric MALT lymphoma, and samples were mainly inpatients rather than outpatients. It is speculated that for indolent MALT lymphoma, patients with *Helicobacter pylori* positive might receive outpatient anti-Helicobacter pylori treatment, and there is no need for further hospitalization if their symptoms were greatly improved. Hussell *T* et al. [8] found that the incidence of HLA-DQA1×0103 and HLA-DQB1×0103 alleles DQA1×0103-DQB1×0601 haplotypes increased in patients with gastric MALT lymphoma. The eradication of *Helicobacter pylori* is the first-line treatment for gastric MALT lymphoma, and the conventional treatment scheme is “quadruple anti-Helicobacter pylori” treatment, that is, PPI + bismuth + two antibiotics, with 10–14 days of treatment. For patients with early-stage focal gastric MALT lymphoma who do not see improvement in anti-Helicobacter pylori treatment, low-dose radiotherapy may be an option, which may preserve gastric function effectively, avoid surgical resection and improve patients' quality of life. For advanced patients (distant lymph node metastasis) or patients with diffuse large B-cell transformation, systematic chemotherapy may be an option. Since there is no standard regimen, patients can choose CHOP or CVP as the primary treatment. For serious complications such as gastrointestinal bleeding and perforation, if endoscopic and medical treatment fail to improve symptoms, patients can choose surgical treatment.

#### 3.5.4. Primary Gastric Diffuse Large B-cell Lymphoma

In this study, there were 24 cases of primary gastric diffuse large B-cell lymphoma, accounting for about 80%. This is the most common type of gastric lymphoma, which can be a new diffuse large B-cell lymphoma or a transformation from gastric MALT lymphoma, but the transformation of gastric MALT lymphoma is relatively rare. Some studies have confirmed that *Helicobacter pylori* infection is the primary risk factor for gastric non-Hodgkin's lymphoma. It is believed to play a key role in the pathogenesis of MALT, but it may also play a role in the development of gastric diffuse large B-cell lymphoma [9]. The primary treatment is CHOP and rituximab. Rituximab binds specifically to the antigen CD20, playing a great role in inhibiting disease recurrence [10]. At present, there is no clear evidence suggesting that *Helicobacter pylori* infection is related to the prognosis of gastric diffuse large B-cell lymphoma. Cheng et al. [11] pointed out that positive *Helicobacter pylori* infection in patients newly diagnosed with primary diffuse large B lymphoma may indicate a good prognosis, whereas negative *Helicobacter pylori* detection may suggest poor prognosis. Eradication of *Helicobacter pylori* has great benefits for patients with primary diffuse large B lymphoma associated with *Helicobacter pylori* infection.

#### 3.5.5. Primary Mantle Cell Lymphoma

In this study, there was only one case of primary mantle cell lymphoma, which is relatively rare. Mantle cell lymphoma accounts for 6% of all non-Hodgkin's lymphoma (NHL). The most common manifestation of mantle cell lymphoma is enlarged lymph nodes, often accompanied by systemic symptoms. Compared with other types of lymphoma, its prognosis is poor. Mantle cell lymphoma often occurs in lymph nodes, and the gastrointestinal tract is the most common site of extranodal lymphoma. At present, immunochemotherapy and autologous stem cell transplantation are the first-line treatment for mantle cell lymphoma. However, this type of treatment is prone to recurrence, and continuous treatment may be required for most patients. To explore the treatment of recurrent gastric mantle cell lymphoma, Toby A. Eyre et al. [12] carried out relevant studies which proved the fast application of anti-CD19 CAR T-cell therapy in this field, the effectiveness of homologous stem cell transplantation, and the application of new therapies such as non-covalent and reversible BTK inhibitors, ROR1 antibody-drug conjugates and bispecific antibodies.

#### 3.5.6. Primary Small Intestinal Lymphoma

Small intestinal lymphoma is one of the malignant tumors of the small intestine, which mostly occurs in ileum, with a high malignant degree and is a rare disease. Patients with small intestinal lymphoma have no obvious symptoms of the disease in the early stage of diagnosis, but most patients may suffer from dull abdominal pain, irregular fever and diarrhea in the late stage. Abdominal mass can be detected during abdominal palpation and there are no obvious enlarged lymph nodes. The pathological type of primary small intestinal lymphoma is mainly non-Hodgkin's lymphoma with a medium and high grade of malignity, which is mainly derived from B cells. It can be roughly divided into small intestinal MALT lymphoma, small intestinal diffuse large B-cell lymphoma, small intestinal mantle cell lymphoma, small intestinal Burkitt lymphoma, small intestinal follicular lymphoma, small intestinal NK/T-cell lymphoma, etc.

#### 3.5.7. Small Intestinal Diffuse Large B-cell Lymphoma

In this study, there were 9 cases of small intestinal diffuse large B-cell lymphoma, accounting for about 50%. At present, a combination of CHOP and rituximab is the primary treatment for small intestinal diffuse large B-cell lymphoma.

#### 3.5.8. Small Intestinal NK/T Cell Lymphoma

In this study, there were 7 cases of small intestinal NK/T-cell lymphoma, accounting for about 38.8%, and all the lesions of NK/T-cell lymphoma were found in the small intestine. NK/T-cell lymphoma is a malignant tumor of the lymphatic system originated from mature NK/T cells. As NK cells and T cells share the same progenitor cells, they have similar functions and expressions of some antigens. NK/T-cell lymphoma is named because it originated from these two types of cells. The incidence of NK/T-cell lymphoma in China and other Asian regions is higher than that in the West, with gastrointestinal NK/T-cell lymphoma being more prone to bleeding and perforation. Compared with B-cell lymphoma, this type of lymphoma has a poor prognosis. NK/T-cell lymphoma occurs most commonly in the nose, less commonly in the gastrointestinal tract. Modified lymphoma is closely related to EB virus infection. All cases of NK/T-cell lymphomas in this study were found in the small intestine.

#### 3.5.9. Small Intestinal Follicular Lymphoma

In this study, there was one case of small intestinal follicular lymphoma. Follicular lymphoma is an indolent B-cell tumor derived from follicular germinal center cells. This type of disease has a long course, and clinical manifestations and prognosis of some patients may have obvious heterogeneity. Such disease is prone to recurrence, with poor prognosis and rapid development. At present, immunochemotherapy is the first-line treatment for small intestinal follicular lymphoma, with rituximab as the most common immunotherapy. Since its introduction, anti-CD20 monoclonal antibody (Rituximab) has reshaped the treatment of follicular lymphoma (FL). Studies by Christian Buske and other scholars [13] show that CT-P10, a generic drug of rituximab, is similar to rituximab in therapeutic effect and drug safety, and its cost is relatively low.

#### 3.5.10. Small Intestinal B-Lymphoblastic Lymphoma

In this study, there was a case of B-lymphoblastic lymphoma, a 29-year-old male with immunohistochemistry as “CK (-), LCA (+), CD3 (-), CD20 (-), CD79a (+), CD10 (+), CD21 (-), CD23 (-), PAX-5 (+), Bcl-2 (+), Ki-67 (+, about 75%), CD5 (-), CD38 (+), CD138 (-), CD34 (+) and Cyclin D1 (-)”. B-lymphoblastic Lymphoma is very invasive. In WHO classification, this type of lymphoma is classified with precursor B-cell lymphoblastic leukemia as class 1 and treated as leukemia. NehaKumari et al. [14] reported a case of B-lymphoblastic lymphoma with pancreatic involvement. After receiving rituximab plus CVAD chemotherapy, the patient showed a good prognosis.

#### 3.5.11. Primary Ileocecal and Colorectal Lymphoma

In this study, 6 cases of ileocecal region and 3 cases of colon were diffuse large B-cell lymphoma. Anatomically, the ileocecal region is part of the colon. Colorectal lymphoma originates from lymphoid reticular tissue, including primary extranodal lymphoma and secondary lymphoma. The former is mostly found in ileocecal region, while the latter is often found in the rectum and sigmoid colon. The incidence of this disease is low, and men are more prone to such disease than women. Surgery is the key treatment for such disease, and patients who undergo a complete radical excision have a better prognosis. Colorectal lymphoma mainly includes MALT lymphoma, mantle cell lymphoma and diffuse large B-cell lymphoma, and follicular lymphoma and T-cell lymphoma. Diffuse large B-cell lymphoma is the most common tissue subtype, followed by mucosa-associated lymphoid tissue (MALT) lymphoma. More than 70% of colorectal lymphomas are proximal to the hepatic flexure [15]. The most common presenting symptoms in patients with colorectal lymphoma are abdominal pain and weight loss. Studies have shown that compared with Western countries, Asia (such as China) usually has higher rates of T-cell lymphomas, which may be due to the difference of host response or the change of etiological factors [15].

## 4. Discussion

This study delved into the incidence types of primary gastrointestinal lymphoma. The data of 78 patients were all retrieved from confirmed cases in the PET/CT center, and the data of 56 patients with pathological results were all retrieved from the inpatient system. In this study, there were no patients with primary intestinal Hodgkin's lymphoma. Primary intestinal Hodgkin's lymphoma has a poor prognosis, with a reported mortality rate of 45–60% within one year after diagnosis. There were no cases of small intestinal MALT lymphoma in this study. The studies of CatherineThieblemont, EmanueleZucca [16] show that small intestinal MALT lymphoma is prone to occur in the Middle East. Primary intestinal Hodgkin's lymphoma has a poor prognosis, with a reported mortality rate of 45–60% within one year after diagnosis. There were no cases of small intestinal MALT lymphoma in this study. The studies of CatherineThieblemont, EmanueleZucca [15] show that small intestinal MALT lymphoma is prone to occur in the Middle East. For small intestinal MALT cases in western countries, it is often related to immigrants in the Middle East. In addition, this lymphoma can be treated with antibiotics (such as tetracycline or metronidazole and ampicillin for at least 6 months), which brings lasting remission to most patients. It is now widely believed that *Campylobacter* jejuni may be related to the pathogenesis of this disease. There was no case of colorectal MALT lymphoma in this study. It is believed that colorectal MALT lymphoma is not related to *Helicobacter pylori*, and it has not been proved that eradication of *Helicobacter pylori* can enhance the curative effect of colorectal lymphoma [17]. However, Takayuki Matsumoto et al. [18] reported a case of rectal MALT, in which after confirming the existence of *Helicobacter pylori*, the patient was treated with eradication of *Helicobacter pylori*, and the condition of rectal MALT lymphoma improved. There are many types of primary gastrointestinal lymphoma. Diffuse large B-cell lymphoma is the most common pathological type of primary gastrointestinal lymphoma, followed by MALT lymphoma. The gastrointestinal tract is the passageway of the digestive system that connects human beings with the outside world. The development of endoscopic technology has greatly benefited the identification of primary gastrointestinal lymphoma. Additionally, gastrointestinal microorganisms such as *Helicobacter pylori*, *Campylobacter* jejuni and Epstein-Barr virus are also related to the occurrence of gastrointestinal lymphoma.

## Figures and Tables

**Figure 1:** Gender distribution of primary gastrointestinal lymphoma.

**Figure 2:** Age distribution of primary gastrointestinal lymphoma.

**Figure 3:** Sites of incidence of primary gastrointestinal lymphoma.

**Figure 4:** Classification of cell origin of primary gastrointestinal lymphoma.

**Figure 5:** Pathological classification of primary gastric lymphoma.

**Figure 6:** Pathological classification of primary small intestinal lymphoma.

## Data Availability

The datasets used and analyzed during the current study are available from the corresponding author on reasonable request.
